# Long-Time Analysis of a Time-Dependent SUC Epidemic Model for the COVID-19 Pandemic

**DOI:** 10.1155/2021/5877217

**Published:** 2021-10-28

**Authors:** Youngjin Hwang, Soobin Kwak, Junseok Kim

**Affiliations:** Department of Mathematics, Korea University, Seoul 02841, Republic of Korea

## Abstract

In this study, we propose a time-dependent susceptible-unidentified infected-confirmed (tSUC) epidemic mathematical model for the COVID-19 pandemic, which has a time-dependent transmission parameter. Using the tSUC model with real confirmed data, we can estimate the number of unidentified infected cases. We can perform a long-time epidemic analysis from the beginning to the current pandemic of COVID-19 using the time-dependent parameter. To verify the performance of the proposed model, we present several numerical experiments. The computational test results confirm the usefulness of the proposed model in the analysis of the COVID-19 pandemic.

## 1. Introduction

Coronavirus disease 2019 (COVID-19) is the infectious disease caused by the most recently discovered coronavirus, which had not been previously identified. Many people infected with the coronavirus have mild to moderate respiratory problems and are naturally recovered without special treatment. However, the older people and patients with underlying medical conditions such as diabetes, cardiovascular, and chronic respiratory diseases are more likely to cause serious complications [1]. The serious problem with COVID-19 is that there are asymptomatic (if symptoms are very mild or no symptoms are identified) infections, and the time from infection to the moment symptoms start is on average 5-6 days and ranges from 1 to 14 days. Because the most common symptom of COVID-19 is fever [2], body temperature measurement is used as a means of detecting infection with COVID-19. Therefore, if an infected person is asymptomatic or does not start showing symptoms, it is difficult to determine whether an infected person is infected, and in this situation, the rate of spread of COVID-19 can be significantly increased. The authors of [3] use a susceptible-infected-recovered (SIR) model and machine learning to simulate the spread of COVID-19 in various scenarios. In order to effectively reduce the scale of the epidemic, it is essential to find and isolate the infected as soon as possible.

Figure 1 shows the sum of the global infected population using country-specific infected population data published by the World Health Organization (WHO) [4]. We can observe the rapid increase in the number of confirmed infections worldwide. If the number of COVID-19 infections continues to rise, many people will die, and the disease will cause enormous economic damage. Therefore, to predict the number of future COVID-19 infections and prepare a prevention and intervention plan in advance, it is important to estimate the unidentified infected cases. If we can estimate the number of unidentified infections using the method proposed in [5], it could help reduce the number of infected cases by evaluating various countries' COVID-19 intervention strategies and adopting effective national intervention strategies.

The SIR model is one of the simplest and most robust models of infectivity. In the traditional SIR model, *β* and 1/*γ* represent the average number of random contacts that an individual has per unit time and the average time for an infected individual to recover, respectively. The traditional SIR model uses constant *β* and *γ* and therefore represents only simple characteristics for infectious diseases [6–8]. The model with constant parameter does not reflect external factors that have a sharp impact on the change of the patient's confirmation criteria or the national prevention policy. Recently, to resolve this problem, a study on the SIR model using *β* and *γ* as time-dependent parameters was conducted, and these research results showed more accurate results for epidemic prediction than before [6, 7].

The SIR model is variously modified and used to analyze infectious diseases. Some researchers analyzed the spread of COVID-19 using a new, nonmonotonous SIR model rather than a monotonous SIR model, in which all susceptible populations are infected and then recovered [9]. In addition, the fractional-order epidemic model has a memory effect and thus has a positive effect on epidemiologic modeling; thus, the researchers developed a fractional-order susceptible-exposed-infected-recovered-deaths (SEIRD) model [10] and a susceptible-infected-recovered-deaths (SIRD) model including multiple fractional features [11]. Some of the other researchers analyzed epidemics and suggested solutions to end them. The researchers compared and analyzed data from multiple countries using a simple SIRD model to show that cultural factors have a great influence on the infection rate in each country and used the modified SIRD model to analyze the epidemics in each country and suggest solutions [12]. Recently, as research on machine learning has become more active, epidemic prediction and analysis using machine learning are also being actively studied. Researchers used the SIR model and machine learning to develop the epidemic model that provide smart healthcare for prediction and prevention of COVID-19 [3]. Nonlinear neural network for predicting COVID-19 cases has been developed [13]. More researchers modify or develop epidemic models to end COVID-19.

The main purpose of this paper is to propose a modified susceptible-unidentified infected-confirmed (SUC) model for long-time analysis of infectious diseases, such as COVID-19, where unconfirmed infections must be considered.

The outline of this paper is as follows.  Section 2 proposes a time-dependent susceptible-unidentified infected-confirmed (tSUC) model. In Section 3, the computational solution algorithm is presented. In Section 4, the computational experiments are performed. Discussion of various infectious disease models and methods of confirming infection of infectious diseases can be found in Section 5. Conclusions are given in Section 6. In addition, the MATLAB source code is given in Appendix for the interested readers.

## 2. Proposed tSUC Epidemic Model

In this paper, we present the tSUC epidemic model for the COVID-19 pandemic, which has a time-dependent transmission parameter. Let *S*(*t*) be the susceptible; *U*(*t*) be the unidentified infected; *C*(*t*) be the confirmed; *β*(*t*)(≥0) be a transmission variable; and *γ* (≥0) be the average number of days taken before the unidentified infected are confirmed. Then, *U*(*t*) is the population where *S*(*t*) is infected with COVID-19 and has no confirmed infection, and *C*(*t*) is the state where *U*(*t*) is confirmed to be infected and no longer spreads the disease. Therefore, *S*(*t*) is infected by *β*(*t*)*S*(*t*)*U*(*t*)/*N* and decreased, *U*(*t*) is increased by *β*(*t*)*S*(*t*)*U*(*t*)/*N*, *C*(*t*) is increased by *γU*(*t*) as confirmed infections, and *U*(*t*) is decreased by *γU*(*t*). Therefore, the derivative of each parameter with respect to time is

(1) $$\begin{array}{c} \frac{\text{d}S\left(t\right)}{\text{d}t}=-\beta \left(t\right)\frac{S\left(t\right)U\left(t\right)}{N}, \end{array}$$

(2) $$\begin{array}{c} \frac{\text{d}U\left(t\right)}{\text{d}t}=\beta \left(t\right)\frac{S\left(t\right)U\left(t\right)}{N}-\gamma U\left(t\right), \end{array}$$

(3) $$\begin{array}{c} \frac{\text{d}C\left(t\right)}{\text{d}t}=\gamma U\left(t\right). \end{array}$$

The unidentified infected population can spread the disease and has not yet been confirmed. The parameter *β*(*t*) is a time-dependent transmission variable, but 1/*γ* is constant as the average number of days taken before the unidentified infected are confirmed. We assume the total population *N* is constant. We note that if *β*(*t*) is constant, then the tSUC model becomes the SUC model [14].  Figure 2 shows schematic illustrations of differently classified groups of the standard SIR and proposed tSUC models. Individuals belonging to *S*, *I*, and *R* groups in the SIR model are susceptible, infected, and recovered, respectively, as shown in the top row of Figure 2. We can subclassify *I* as UI and CI which are unconfirmed-infected and confirmed-infected, respectively; see the middle row of Figure 2. In the tSUC model, *U* is UI and *C* is CI ∪ *R* (see the bottom row of Figure 2).

In the standard SIR model, *γ*_SIR_ is the reciprocal of the period during which an infected individual acquires antibodies and heals. However, in the proposed tSUC model, *γ*_SUC_ is the reciprocal of the period during which an unidentified infected individual can spread an infectious disease until the infection is confirmed. Generally, 1/*γ*_SIR_ is larger than 1/*γ*_SUC_ (see Figure 3).

## 3. Numerical Solution Algorithm

The tSUC model can be solved by a fourth-order Runge–Kutta (RK4) method. First, let us rewrite equations (1)–(3) as follows:

(4) $$\begin{array}{c} \frac{\text{d}S\left(t\right)}{\text{d}t}=f\left(\beta \left(t\right),S\left(t\right),U\left(t\right)\right),\\ \frac{\text{d}U\left(t\right)}{\text{d}t}=g\left(\gamma ,\beta \left(t\right),S\left(t\right),U\left(t\right)\right),\\ \frac{\text{dC}\left(t\right)}{\text{d}t}=h\left(\gamma ,U\left(t\right)\right),\\ S\left(t_{0}\right)=S_{0},\;U\left(t_{0}\right)=U_{0},\;C\left(t_{0}\right)=C_{0}. \end{array}$$

Second, let *S*_*n*_=*S*(*n*Δ*t*), *U*_*n*_=*U*(*n*Δ*t*), and *C*_*n*_=*C*(*n*Δ*t*), where Δ*t* is a time step. For *n*=0,  1,  2,…, we have the following discrete equations:

(5) $$\begin{array}{c} S_{n+1}=S_{n}+\frac{1}{6}\Delta t\left(k_{11}+2k_{12}+2k_{13}+k_{14}\right), \end{array}$$

(6) $$\begin{array}{c} U_{n+1}=U_{n}+\frac{1}{6}\Delta t\left(k_{21}+2k_{22}+2k_{23}+k_{24}\right), \end{array}$$

(7) $$\begin{array}{c} C_{n+1}=C_{n}+\frac{1}{6}\Delta t\left(k_{31}+2k_{32}+2k_{33}+k_{34}\right), \end{array}$$

(8) $$\begin{array}{c} t_{n+1}=t_{n}+\Delta t, \end{array}$$

and *γ*,  *β*_*n*_,  and *U*_0_ are the unknown parameters. To solve the discrete system of equations (5)–(7), we need to know these parameter values. However, in the real-world population, *β*, *γ*, and the number of the unidentified infected cases *U* are unknown; and only the number of cumulative confirmed cases *C* is known. To estimate the unknown unidentified infected cases *U*, we use the tSUC model and the fitting function **lsqcurvefit** in MATLAB R2021a, which is a nonlinear curve-fitting solver in a least-squares sense [15].

### 3.1. Data Smoothing

As a preprocessing of the epidemic data, we take 7-day average data because the number of testing COVID-19 is different day by day. First, the number of new confirmed cases (Δ*C*) is calculated using the number of cumulative confirmed cases as follows: $\Delta C_{i}={\hat{C}}_{i+1}-{\hat{C}}_{i},\;i=1,2,\ldots ,p-1$, where *p* is the number of the given real cumulative confirmed cases ${\hat{C}}_{i}\;\left(i=1,2,\ldots ,p\right)$. Second, we calculate the 7-day simple moving average of the number of new confirmed cases. Δ_ave_*C*_*i*_=(Δ*C*_*i*_+Δ*C*_*i*+1_+⋯+Δ*C*_*i*+6_)/7,  *i*=1,2,…, *p* − 7. Finally, the smoothed cumulative confirmed case data ref*C* are generated using the 7-day simple moving average of new confirmed cases as follows:

(9) $$\begin{array}{c} C_{i}^{\text{ref}}={\hat{C}}_{7}+\sum_{j=1}^{i}\Delta_{\text{ave}}C_{j},\;i=1,2,\ldots ,p-7. \end{array}$$

### 3.2. Estimating Parameters

Let *β*=[*β*_*n*_1__, *β*_*n*_2__,…, *β*_*n*_*L*__] be the vector with sample transmission values at sample points **t**=[*t*_*n*_1__, *t*_*n*_1__+*q*, *t*_*n*_1__+2*q*,…, *t*_*n*_*L*__], where *q* is a sampling interval, *t*_*n*_1__ is the starting day, and *t*_*n*_*L*__ is the last check day, which will be less than or equal to the end day of the case data.

Using the piecewise interpolation, we can obtain values at between *t*_*n*_1__ and *t*_*n*_*L*__. We obtain optimal parameters *γ*,  *β*,  *U*_0_ which minimize the following cost function:

(10) $$\begin{array}{c} E\left(\gamma ,\;\beta ,\;U_{0}\right)=\frac{1}{2}\sum_{i=1}^{p-7}{\left(C_{i}^{\text{ref}}-C_{n_{i}}\right)}^{2}, \end{array}$$

where *C*_*n*_*i*__(*i*=1,2,…, *p* − 7) are the numerical solutions from equations (4) to (6) at the corresponding times. We compute the optimal parameter values of (*γ*,  *β*,  *U*_0_) that minimize the cost function as

(11) $$\begin{array}{c} \left[\gamma ,\;\beta ,\;U_{0}\right]=lsqcurvefit\left('\text{tSUCmodel}{}^{\prime },\left[\gamma^{0},\;\beta^{0},\;U_{0}^{0}\right],T\;da\;ta,C\;da\;ta,lb,ub\right), \end{array}$$

where [*γ*,  *β*,  *U*_0_] are the optimized parameters and [*γ*,  *β*^0^,  *U*_0_^0^] are the initial guess of parameters for the tSUCmodel, **C**  **da**  **ta** is the real cumulative confirmed case data at times **T**  **da**  **ta**, lb is the lower bound, and ub is the upper bound.

## 4. Numerical Tests

### 4.1. Convergence and Stability Tests

In this section, to verify the accuracy of the proposed algorithm, we perform a convergence test. We generate a reference solution using the following initial data: *N*=300000, *C*_0_=20000, *U*_0_=2000, *γ*=1/4, and *β*(*t*)=0.3+0.1*t*.  Table 1 shows that the proposed method has fourth-order accuracy. Here, the following definitions are used: Δ*t*=2^−2^, the final time *T*=4, *l*_2_-error $=\sqrt{{\left(S^{\text{ref}}-S_{N_{t}}\right)}^{2}+{\left(U^{\text{ref}}-U_{N_{t}}\right)}^{2}+{\left(C^{\text{ref}}-C_{N_{t}}\right)}^{2}}$, and *N*_*t*_=*T*/Δ*t*, where we use the reference solutions *S*^ref^,  *U*^ref^,  *C*^ref^ computed with sufficiently small Δ*t*^ref^=2^−10^.

Next, we numerically test the stability of the tSUC model. Figures 4(a)–4(c) show the computational results for *S*, *U*, and *C*, respectively. The results are obtained using Δ*t*=0.1, 1,10 and *β*(*t*)=0.3+0.1*t*/*T* up to time *T*=30. The proposed algorithm shows that it has nonnegative solutions even with large time steps.

### 4.2. Simulation on Real Data

For all simulations, it is assumed that the time step size Δ*t*=0.1, *β* and *U*_0_ are positive real numbers, and the upper and lower bound of *γ* are 1 and 1/14, respectively. Because *γ* is the reciprocal of the average time until an unidentified infected person is confirmed, it can be inferred from the period of symptom onset and epidemiological investigation. In this section, simulations are performed to confirm that the proposed method can estimate the optimal parameters for estimating the change in the number of unidentified infected cases over a long period of time and the change in the number of new confirmed cases using actual confirmed cases. First, data smoothing is performed on actual confirmed cases for parameter estimation. The actual confirmed case data and smoothed actual confirmed case data are called *C*^raw^ and *C*^ref^, respectively.  Figure 5 shows *C*^raw^ and *C*^ref^ from March 2, 2020, to July 23, 2021, in the Republic of Korea [4].

Next, we estimate the parameters beta and gamma using smoothed *C*_*i*_^ref^(*i*=1,2,…, 502) and the following initial conditions: *γ*^0^=1/4, *β*^0^=[1/3,…, 1/3], and *U*_0_=2(*C*_2_^ref^ − *C*_1_^ref^)=771.71.

Figure 6 shows time-dependent *β*(*t*) when *q*=60.

In equation (2), the rate of change of *U* is dependent on the values of *β*(*t*)*S*/*N* − *γ*. If *β*(*t*)*S*/*N* − *γ* is positive, then *U* increases, and if *β*(*t*)*S*/*N* − *γ* is negative, then *U* decreases.  Figure 7 shows the change in the estimated value according to *q*. In Figure 7(c), we can observe that the value of estimated *β*(*t*)*S*/*N* − *γ* according to *q* is different. When *q* is 2, the number of checkpoints is very large, resulting in overfitting. When *q* is 30, the number of checkpoints is relatively small, showing simple characteristics. Therefore, we need to use appropriate *q*.

We use *q*=7 to characterize the epidemic in detail without overfitting.  Figure 8 shows the calculated results. It can be observed that the estimated parameters represent the characteristics of the epidemic in detail, and the *β*(*t*)*S*/*N* − *γ* values represent the changes in the new confirmed cases.

## 5. Discussion

In this section, we discuss the advantages and disadvantages of the proposed method and future work. We proposed the tSUC model which enables us to analyze long-time analysis; thus, it is possible to estimate changes in the number of unidentified infected cases over a long period of time and the transmission over time and to estimate the number of unidentified infected cases in the present and past. If we can estimate the number of unidentified infected cases and its long-time trend, then we can plan and prepare the number of testing stations for COVID-19 testing, quarantine policies according to the transmission, and incentives for COVID-19 testing and vaccines. However, limitations of the proposed model are that it cannot represent changes in detailed factors such as vaccines or cultural factors, and it does not consider birth and death. The proposed model uses the least-squares method because it is simple and easy to use. However, if a fitting function such as a deep learning neural network is used, more effective results can be obtained for predicting the future [13].

The fractional-order epidemic model for the proposed model has a memory effect because it uses past history; thus, we think it is a more effective method for epidemic models such as COVID-19 with an incubation period [10, 11]. The proposed model is affected by the period during which infection of an unidentified infected person is confirmed. The method of confirmation of COVID-19 infection with X-ray images by the hybrid model using the deep learning technique can confirm the infection quickly, simply, and accurately [16]. Therefore, we consider the following future work. First, we use deep learning neural networks to solve the tSUC model to analyze infectious diseases such as COVID-19 and predict the future. Second, we propose a model specialized for infectious diseases with an incubation period by modifying it to the fractional order of the proposed model. Finally, we propose a modified tSUC model that considers birth and death.

## 6. Conclusion

We proposed a long-time analysis of a tSUC model for the COVID-19 pandemic. The parameters of an epidemic model are important indicators of the characteristics of an epidemic. The parameters of an epidemic model change over time due to several factors. Therefore, estimating epidemic parameters and fixing them as a single value can represent only simple characteristics; also, it is difficult to express detailed characteristics or long-time analysis. To solve the problem of time-varying epidemic parameters, one of the parameters can be made time-dependent to estimate the optimal parameters for long-time epidemic analysis, allowing detailed characterization of epidemics over time. We demonstrated the effectiveness of the proposed method by estimating epidemic parameters using real data and performing several tests to confirm that the estimated parameters are characteristics of real data. It can be confirmed that the parameters estimated from the numerical results are suitable for long-time analysis of the epidemic, and detailed data analysis can be performed in the long term than the methods used in the existing SUC model studies.

## Figures and Tables

**Figure 1:** Number of populations infected with COVID-19 worldwide.

**Figure 2:** Schematic diagram of the standard SIR and proposed tSUC model.

**Figure 3:** Schematic diagram for 1/*γ* of the standard SIR and proposed tSUC models.

**Figure 4:** (a) Susceptible cases. (b) Unidentified infected cases. (c) Confirmed cases.

**Figure 5:** Raw confirmed data and confirmed data smoothed by the proposed method: (a) confirmed cases and (b) new confirmed cases.

**Figure 6:** Schematic diagram of time-dependent *β*(*t*) when *q*=60 of the proposed method.

**Figure 7:** Numerical solutions: (a) confirmed cases, (b) new confirmed cases, and (c) calculated results.

**Figure 8:** Numerical solutions: (a) confirmed cases, (b) new confirmed cases, (c) unidentified infected cases, and (d) calculated results.

**Table 1:** *l*_2_-norm error and convergence rates with various Δ*t*.

Case	Δ*t*	Rate	Δ*t*/2	Rate	Δ*t*/4	Rate	Δ*t*/8
*l*_2_-error	3.0679*e *− 3	3.98	1.9458*e *− 4	3.99	1.2243*e *− 5	4.00	7.6600*e *− 7

## Data Availability

The data used to support the findings of this study are included within the article.

## Appendix

The following code is the main program, which is available from the corresponding author's web page (https://mathematicians.korea.ac.kr/cfdkim/open-source-codes/).

  clear all; close all; clc; global N C0 checkTime.
  datatable = readtable('WHO_Korea_data.xlsx');
  Daydata = datatable{:,1}; OriCdata = datatable{:,6};
  sp = 60; ep = 568; *p* = ep-sp+1;
  refTdata = [1:p]; NewTdata = [2:p]; Tdata = [8:p]; *N* = 5.0*e*+7;
  for *i* = 1:p.
  rawC(*i*) = OriCdata(sp-1+*i*);
  end.
  rawdC = diff(rawC);
  for *i* = 1:p-7.
  refdC(*i*) = mean(rawdC(*i*:*i*+6));
  refC(*i*) = rawC(7) + sum(refdC(1:i));
  end.
  Cdata = refC;
*q* = 7;
  checkTime = unique([Tdata(1):q:Tdata(end) Tdata(end)]);
  g0 = 1/4; *b*0 = 1/3∗ones(length(checkTime),1);
*U*0 = 2.0∗(Cdata(2)-Cdata(1)); *C*0 = Cdata(1);
  param = lsqcurvefit(@tSUCmodel, [g0; b0; U0; ], [Tdata], [Cdata],….
  [1/14; 0∗b0; 0∗U0; ], [1]);
*g* = param(1); U(1) = param(end); C(1) = C0; S(1) = N–C(1)-U(1);
*T* = length(Tdata)-1; dt = 0.1; Nt = round(T/dt);
*t* = linspace(Tdata(1),Tdata(end),Nt+1);
*b* = interp1(checkTime, param(2:end-1),t,'pchip');
*F* = @(b,S,U) -b∗S∗U/N; *G* = @(g,b,S,U) b∗S∗U/N-g∗U; *H* = @(g,U) g∗U;
  for *i* = 1:Nt.
  k11 = F(b(*i*),S(*i*),U(*i*));
  k21 = *G*(g,b(*i*),S(*i*),U(*i*));
  k31 = H(g,U(*i*));
  k12 = F((b(*i*)+*b*(*i*+1))∗0.5,S(*i*)+0.5∗dt∗k11,U(*i*)+0.5∗dt∗k21);
  k22 = *G*(g,(b(*i*)+*b*(*i*+1))∗0.5,S(*i*)+0.5∗dt∗k11,U(*i*)+0.5∗dt∗k21);
  k32 = H(g,U(*i*)+0.5∗dt∗k21);
  k13 = F((b(*i*)+*b*(*i*+1))∗0.5,S(*i*)+0.5∗dt∗k12,U(*i*)+0.5∗dt∗k22);
  k23 = *G*(g,(b(*i*)+*b*(*i*+1))∗0.5,S(*i*)+0.5∗dt∗k12,U(*i*)+0.5∗dt∗k22);
  k33 = H(g,U(*i*)+0.5∗dt∗k22);
  k14 = F(b(*i*+1),S(*i*)+dt∗k13,U(*i*)+dt∗k23);
  k24 = *G*(g,b(*i*+1),S(*i*)+dt∗k13,U(*i*)+dt∗k23);
  k34 = H(g,U(*i*)+dt∗k23);
  S(*i*+1) = S(*i*)+dt∗(k11 + 2∗k12 + 2∗k13 + *k*14)/6;
  U(*i*+1) = U(*i*)+dt∗(k21 + 2∗k22 + 2∗k23 + *k*24)/6;
  C(*i*+1) = C(*i*)+dt∗(k31 + 2∗k32 + 2∗k33 + *k*34)/6;
  end.
  dC = diff(C(1 : Nt/(length(Tdata)-1):end));
figure 1; hold on; box on;
  plot(Tdata, Cdata,'k--'); plot(t,C); title('Confirmed cases')
figure 2; hold on; box on;
  plot(Tdata(2:end),refdC(2:end),'k--'); plot(Tdata(2:end),dC);
  title('New Confirmed cases')
figure 3; hold on; box on;
  plot(Tdata(2:end),dC/g,'k--'); plot(t,U);
  title('Unidentified infected cases')
figure 4; hold on; box on;
  plot(t,(b.∗S)/N-g); yline(0,'--'); title('∖beta(S/N)-∖gammaˆ{∖prime})
  function *f* = tSUCmodel(Parameter, Tdata).
  global N C0 checkTime;
*g* = Parameter(1); U(1) = Parameter(end); C(1) = C0;
  S(1) = N–C(1)-U(1); *T* = length(Tdata)-1; dt = 0.1; Nt = round(T/dt);
*t* = linspace(Tdata(1),Tdata(end),Nt+1);
*b* = interp1(checkTime, Parameter(2:end-1),t,'pchip');
*F* = @(b,S,U) -b∗S∗U/N; *G* = @(g,b,S,U) b∗S∗U/N-g∗U; *H* = @(g,U) g∗U;
  for *i* = 1:Nt.
  k11 = F(b(*i*),S(*i*),U(*i*));
  k21 = *G*(g,b(*i*),S(*i*),U(*i*));
  k31 = H(g,U(*i*));
  k12 = F((b(*i*)+*b*(*i*+1))∗0.5,S(*i*)+0.5∗dt∗k11,U(*i*)+0.5∗dt∗k21);
  k22 = *G*(g,(b(*i*)+*b*(*i*+1))∗0.5,S(*i*)+0.5∗dt∗k11,U(*i*)+0.5∗dt∗k21);
  k32 = H(g,U(*i*)+0.5∗dt∗k21);
  k13 = F((b(*i*)+*b*(*i*+1))∗0.5,S(*i*)+0.5∗dt∗k12,U(*i*)+0.5∗dt∗k22);
  k23 = *G*(g,(b(*i*)+*b*(*i*+1))∗0.5,S(*i*)+0.5∗dt∗k12,U(*i*)+0.5∗dt∗k22);
  k33 = H(g,U(*i*)+0.5∗dt∗k22);
  k14 = F(b(*i*+1),S(*i*)+dt∗k13,U(*i*)+dt∗k23);
  k24 = *G*(g,b(*i*+1),S(*i*)+dt∗k13,U(*i*)+dt∗k23);
  k34 = H(g,U(*i*)+dt∗k23);
  S(*i*+1) = S(*i*)+dt∗(k11 + 2∗k12 + 2∗k13 + *k*14)/6;
  U(*i*+1) = U(*i*)+dt∗(k21 + 2∗k22 + 2∗k23 + *k*24)/6;
  C(*i*+1) = C(*i*)+dt∗(k31 + 2∗k32 + 2∗k33 + *k*34)/6; s.
  end.
*f* = interp1(t,C,Tdata);
  end.
